The article "Magnetic Resonance Imaging Data Features to Evaluate the Efficacy of Compound Skin Graft for Diabetic Foot" was published in 2022. Journal: Contrast Media Mol Imaging.

# Magnetic Resonance Imaging Data Features to Evaluate the Efficacy of Compound Skin Graft for Diabetic Foot

**DOI:** 10.1155/2022/5707231

**Published:** 2022-06-13

**Authors:** Chunlei Wang, Xiaomei Yu, Ying Sui, Junhui Zhu, Bo Zhang, Yongtao Su

**Affiliations:** ^1^Department of Burn Skin Surgery, PKUcare Luzhong Hospital, Zibo 255400, Shandong, China; ^2^Innovation Research Institute, Shandong University of Traditional Chinese Medicine, Jinan 250355, Shandong, China

## Abstract

This study aimed to analyze the role of magnetic resonance imaging (MRI) data characteristics based on the deep learning algorithm in evaluating the treatment of diabetic foot (DF) with composite skin graft. In this study, 78 patients with DF were randomly rolled into the experimental group (composite skin graft) and control group (autologous skin graft) with 39 patients in each group. MRI scans were performed before and after treatment to compare the changes of experimental observation indicators such as healing time, recurrence rate, and scar score. The results showed that T1-weighted imaging (T1WI) of the scanning sequence was considerably increased in the experimental group after treatment. The signal intensity of fat-suppressed T2-weighted imaging (T2WI) and fat-suppressed T1WI enhancement sequences was considerably decreased (*P* < 0.05). In addition, compared with the control group, the recurrence rate, healing time, and scar score in the experimental group were considerably decreased (*P* < 0.05). The accuracy, specificity, and sensitivity of MRI imaging information in evaluating the therapeutic effect of DF patients were 85.2%, 89.75%, and 86.47%, respectively. According to the specificity and sensitivity, the subject operating characteristic curve was drawn, and the area under the curve was determined to be 0.838. In summary, MRI image data characteristics based on the deep learning algorithm can provide auxiliary reference information for the efficacy evaluation of compound skin transplantation for DF.

## 1. Introduction

In recent years, with the rapid growth of the incidence of diabetes, the number of diabetic foot (DF) patients has gradually increased [1]. DF is a very serious complication caused by diabetes, usually manifested as infection of the lower limbs, ulcers, and even the destruction of deep tissue and bone marrow. Pathological changes involve neuropathy and peripheral vascular lesions of the lower limbs. The disease is characterized by a long period of disease, which is often difficult to cure, high treatment cost, and a very high recurrence rate, thus bringing serious burden and harm to patients and families all over the world [2–5]. According to statistics, in 2003, the number of diabetes patients in the world was close to 200 million, while in 2014, the number of diabetes patients has exceeded 400 million. At this rate, the number of diabetes patients in the world will exceed 600 million by 2035 [6–8]. In China, the number of diabetes patients is also increasing rapidly. The literature reported that the incidence of diabetes in China was only 0.67% in 1980. In 2013, the incidence of diabetes has increased to more than 10%, which means that 10-11 out of 100 randomly selected people in China have diabetes. The incidence of DF is also high, and there are about 8 DF patients in every 100 people [9, 10]. Clinical DF is often difficult to cure, and the mechanism is that the DF patients lack growth factors required for normal healing. DF patients increased proteolytic activity, resulting in a rapid increase in matrix metalloproteinase concentration, so that the wound could not heal normally. The function of fibroblasts in patients is limited, resulting in the difficulty of normal synthesis of collagen and abnormal blood vessel formation, resulting in affected wound healing. In DF patients, the normal activity of white blood cells in the body inhibited, and sufficient neutrophils cannot gather around the wound, leading to the failure of the antiinfection function of the wound site and the limitation of blood supply, thus affecting wound healing [11–14].

Slow healing of DF ulcer seriously affects the quality of life of patients. Therefore, the treatment and management of DF patients is particularly important [15].

The treatment of DF mainly includes medical treatment and surgical treatment. First, according to the situation of DF wounds, different methods of debridement and dressing change should be appropriately given to remove local bacteria or infected microorganisms to promote wound healing, and systemic antibiotic treatment should be given to patients at the same time [16, 17]. After long-term conservative medical treatment, the wound will not heal for a long time and even the infection will be aggravated. At that time, it is necessary to use surgical treatment to remove the necrotic limbs, remove the potential infection foci, and avoid the development of DF into sepsis. Skin grafting is an operation with significant efficacy for the repair of large areas of wounds and is a good choice for the healing of diabetic foot wounds [18–20]. Skin grafting is often used to repair DF ulcers in clinical practice. When simple skin grafting is adopted to repair wounds, such as medium or full thickness skin, the survival rate of full thickness skin transplantation is often low due to the existence of granulation wounds. After medium thick skin transplantation, the healing barrier of donor site will be caused, resulting in the generation of new surface. Thick blade skin transplantation can solve the problem of low survival rate. However, due to the lack of dermis after skin grafting, the friction resistance and pressure resistance of the surface are poor, and it is easy to cause secondary ulceration. Composite skin transplantation can solve the above problems. In this study, acellular allogeneic dermal matrix and autologous skin combined with skin grafting were used to treat DF patients. Acellular allogenic dermal matrix refers to the fixation and cross-linking of allogenic skin extracellular matrix with solid agent treatment. Then, chelating agents and trypsin were used to remove the epidermis, and DNA and RNA enzymes and chemical agents were used to treat the reticular acellular allogenic dermis to reduce the cellular immune response [21].

Diabetes can be diagnosed and observed by X-ray, computed tomography (CT), magnetic resonance imaging (MRI), and other influencing methods. X-rays are an economical method and are often used to evaluate bone infection, but changes in the bone usually do not show up until 1-2 weeks after infection. The density resolution of CT is higher than that of X-ray, but compared with MRI, the early changes of the lesions displayed by CT are obviously inferior. MRI and CT examination have the same price, high soft tissue resolution, and spatial resolution, which can diagnose abnormal changes of bone early and can accurately diagnose the range of lesions and whether there is infection, providing a reliable basis for the selection of clinical plans. Therefore, MRI has unique advantages in the diagnosis of DF. There are many imaging features around ulcer skin of DF. Computer vision algorithms can make use of these visual symbols to distinguish and use deep learning-based methods for medical image analysis, and processing has become an important part of imaging diagnosis. It plays a crucial role in detecting a variety of diseases, including DF ulcers. As a target detection algorithm, the single shot detector (SSD) is one of the main target detection frameworks. With high speed and accuracy, it can detect objects on different feature maps at different scales, resist changes in object size to a certain extent, and give more robustness to the network. Methods and technologies based on deep learning have been widely applied in the medical field and have a high clinical application value [22].

In this research, DF patients meeting the requirements were selected and divided into the experimental group and control group. Different methods were used for treatment, and MRI scanning and clinical indicators were observed and compared to comprehensively evaluate the application value of MRI imaging information based on the deep learning algorithm in the curative effect of compound skin transplantation for diabetic foot, so as to provide a feasible plan for the clinical treatment of DF.

## 2. Materials and Methods

### 2.1. The Research Objects

In this study, 78 patients with DF admitted to hospital from January 10, 2018, to May 10, 2020, were selected and divided into the experimental group and control group according to their treatment intention, with 39 patients in each group. Composite skin graft and autologous skin graft were adopted for treatment in the experimental group and control group, respectively. This study had been approved by the ethics committee of hospital, and the patients' families had been informed of this study and signed informed consent.

Inclusion criteria were as follows: patients diagnosed with DF according to diagnostic criteria, patients had been treated with combined skin graft/autologous skin graft, patients older than 18 years, patients who had signed informed consent, and patients with contraindications were not examined.

Exclusion criteria were as follows: patients with other serious underlying diseases, patients with severe allergic constitution, patients with obesity, patients with lower limb amputation, patients whose family members did not agree or sign informed consent, and patients with poor coordination or did not accept follow-up.

### 2.2. Treatment Methods

Patients in the experimental group were treated with compound skin graft. First, debridement was performed to remove the necrotic skin, subcutaneous tissue, tendon, fascia, and necrotic bone. Then, the skin wound was covered with VSD dressing, and the negative pressure sealing drainage technology was used to keep the VSD unobstructed by periodic flushing. VSD was replaced regularly until the necrotic tissue at the depth of the wound was removed and the granulation tissue was fresh and full. For skin grafting, the acellular allogenic dermal matrix prepared was taken and washed with normal saline for three times. The size of the wound was compared and trimmed, not exceeding the edge of the wound. Acellular allogenic dermal matrix was fixed on the wound surface with net face up and dermal face down to make it closely fit without leaving gaps. The skin of the leg was taken with an electric skin knife, transplanted on the wound surface, and fixed. It was washed with normal saline to make it closely fit, leaving no dead cavity. Then, VSD material was covered on the surface again, and negative pressure was applied to seal drainage. The patency of the VSD was checked regularly every day, and the affected limb was kept in a high position. VSD material was removed 7–10 days later, and the survival of skin grafting was observed. Dressing change and nursing were continued on time until the wound healed completely. The control group was treated with autologous skin graft. Autologous skin graft thickness was about 0.4 mm. Other treatments were the same as compound skin graft.

### 2.3. MRI Scan

3.0 T MR imaging scanning instrument was used for scanning. Sagittal plane, transverse plane, and coronal plane scanning were performed according to the lesion site of the foot. Special coil for the foot was adopted. The scanning sequence included T1-weighted Imaging (T1WI), T2-weighted Imaging (T2WI), and fat-suppressed T1WI. Enhancement scan was performed about 3 min after the gadolinium contrast agent was injected. The injection volume was calculated according to 0.1 mmoL/kg, and the injection rate was 2.5 mL/s. Specific scanning parameters are shown in Figure 1.

### 2.4. Deep Learning Algorithm Model

As an excellent target detection model, the single shot detector (SSD) has been widely used. SSD uses feature graphs from multiple convolutional layers to perform boundary box regression and target category prediction. Target detection is carried out at different convolutional layers in combination with features extracted from feature graphs of different sizes, so as to improve the accuracy of detecting small objects in size. The specific flowchart is shown in Figure 2.

The original photos were first input to obtain feature maps of different scales. Four prior frames were set, namely, predetermined frames of the target. Feature maps of different sizes corresponded to prior frames of different sizes. The side length of the smaller prior frame was set as *x*, the side length of the larger prior frame as $\sqrt{x\times d}$, and the aspect ratio as *Ar*. Then, the length (*C*) of the rectangular frame can be expressed by

(1) $$\begin{array}{c} C=\sqrt{Ar}\times x. \end{array}$$

The width (*K*) of the rectangular box is expressed by

(2) $$\begin{array}{c} K=\frac{1}{\sqrt{Ax}\times x}. \end{array}$$

*x* and *d* are determined by

(3) $$\begin{array}{c} M_{0}=Mx+\frac{M\;d-Mx}{s-1}\left(a-1\right). \end{array}$$

The range of *a* is shown in

(4) $$\begin{array}{c} a\in \left[1,s\right]. \end{array}$$

In equation (4), *s* represents the number of feature maps. When *Ar* is 1, a scale will be added, as shown in

(5) $$\begin{array}{c} M_{0}=\sqrt{M_{0}\times M_{0+1}}. \end{array}$$

Based on the average accuracy of the test means in different test sets, the accuracy of SSD ranged from 67.0% to 78.8%. SSD has the dual guarantee of accuracy and detection rate. The algorithm proposes that it has a variety of width-to-height ratio prior frames, which makes it have a good detection effect for all kinds of objects of different sizes.

### 2.5. Evaluation Indexes

Basic data collected from the two groups were compared and analyzed, including age, sex, course of disease, body mass index, and glycosylated hemoglobin (HbAlC), and Wagner grading of DF was performed using MRI scan. According to the overall cardiac function parameters obtained from MRI scans, the changes of T1WI, fat-suppressed T2WI, and enhancement sequences of MRI scans were observed and compared between the two groups to analyze the relationship between MRI intensity signal and therapeutic effect after combined skin graft treatment. The wound healing of patients in the two groups was recorded, and the time from surgical treatment to wound healing was recorded and compared. The total number of cases was *S*, the number of cases was *C*, and the complete healing rate *R* was calculated according to

(6) $$\begin{array}{c} R=\frac{c}{s}\times 100\%. \end{array}$$

The healing time of the donor skin area was recorded and compared. The healing state was determined when the wound surface of the donor skin area was gradually epithelialized, and the skin surface was dry. Scar status was recorded and compared between the two groups. The patients were scored in terms of skin graft softness, color, thickness, and vascular distribution using the Vancouver Scar Scale. For the calculation and statistics of the recurrence rate, the patients were followed up after discharge, and the recurrence rate of the two groups of patients was calculated. The number of patients with reulcer at the same site was denoted as *G*, the total number of patients in each group was denoted as *S*, and the recurrence rate *F* was calculated according to

(7) $$\begin{array}{c} F=\frac{G}{S}\times 100\%. \end{array}$$

In this study, experimental observation results after transplantation treatment were used as the reference standard, and three common indicators were used to evaluate the ability of MRI image data characteristics to evaluate the therapeutic effect of DF patients. Accuracy, specificity, and sensitivity were calculated in the following equations.

(8) $$\begin{array}{c} \text{Accuracy}=\frac{TA+TB}{TA+FC+TB+F\;D}, \end{array}$$

(9) $$\begin{array}{c} \text{Specificity}=\frac{TB}{FC+TB}, \end{array}$$

(10) $$\begin{array}{c} \text{Sensitivity}=\frac{TA}{F\;D+TA}. \end{array}$$

Among them, *TA* is true positive, indicating that the diagnosis result is positive, which is positive. *TB* refers to true negative, indicating that the diagnosis is negative, but negative. *FC* is false positive, meaning that the diagnosis is positive, but negative. *FD* is false negative, which means the actual result is positive and the diagnostic result is negative.

Receiver operating characteristic (ROC) curve was used to represent the ability of MRI image data characteristics to evaluate the therapeutic effect of DF patients. According to ROC, the area under ROC curve (AUC) was determined.

### 2.6. Statistical Methods

All experimental data were statistically analyzed by the SPSS 24.0 software. The measurement data were expressed by mean ± standard deviation ($\bar{x}$ ± *s*), and the counting data were statistically inferred by the *χ*^2^ test. If the measurement data conformed to normal distribution, the *t*-test was adopted. *P* < 0.05 was statistically significant.

## 3. Results

### 3.1. MRI Imaging Results

Figure 3 shows MRI images of different DF patients in different planes.  Figure 3(a) shows a 55-year-old male DF patient who had suffered from diabetes for 11 years with swollen feet and ulcers.  Figure 3(b) shows a DF patient, male, 57 years old, with observed skin continuity interruption, abscess, and sinus tract.  Figure 3(c) shows a DF patient, male, 64 years old, with high blood glucose level for 8 years. Both feet were broken and admitted to hospital for treatment.  Figure 3(d) shows a 63-year-old male DF patient with elevated blood glucose for 13 years, who was hospitalized with foot ulcer and discharge.  Figure 3(e) shows a deep penetrating skin ulcer and sinus tract on the plantar.

### 3.2. SSD Algorithm Target Detection

In Figure 4, the SSD target detection model was used to accurately locate and extract features of wounds requiring skin grafting in MRI images, which was also applicable to target detection with different aspect ratios.

### 3.3. Comparison of Basic Data between the Two Groups

Through comparison, there were no substantial differences in age, gender, course of disease, body mass index, HbAlC, and Wagner grading between the two groups (*P* < 0.05, Figure 5).

### 3.4. Comparison Results of MRI Scanning Sequence Signal

MRI scan sequence signal intensity of patients before and after treatment was obtained. Comparative analysis showed that T1WI signal intensity of the experimental group was considerably increased after treatment, while the signal intensity of fat-inhibited T2WI and fat-suppressed T1WI enhanced sequence was considerably decreased (*P* < 0.05, Figure 6).

### 3.5. Results of Experimental Indicators after Treatment

The results showed that compared with the control group, there was no statistical difference in the wound healing time and complete healing rate in the experimental group (*P* > 0.05), while the recurrence rate, healing time of the donor skin area, and scar score were considerably decreased (*P* < 0.05). The specific results are shown in Figures 7 and 8.

### 3.6. MRI Imaging Information Evaluation Effectiveness

Through calculation of accuracy, specificity, and sensitivity, it was found that MRI imaging information had high accuracy, specificity, and sensitivity in evaluating the therapeutic effect of DF patients, which were 85.2%, 89.75%, and 86.47%, respectively. ROC curves were drawn based on MRI imaging information to evaluate the specificity and sensitivity of therapeutic effects in DF patients (Figure 9). Meanwhile, AUC was determined to be 0.838 according to ROC.

## 4. Discussion

At present, the number of patients with diabetes is increasing. As one of the most serious complications of diabetes, DF brings serious economic and mental burden to patients and their families. It is estimated that the number of diabetes patients in the world will exceed 600 million in 2035. DF has a long disease cycle, difficult to cure, high treatment cost, and high recurrence rate. Studies reported that every 20 seconds, a DF patient faces amputation, which seriously affects the quality of life of the patient, and the 5-year mortality rate of the patient after amputation is more than 50%. Therefore, the timely treatment and management of DF patients is crucial [23]. Skin grafting can help DF patients repair ulcers. Skin grafting alone often leads to the low survival rate of full thickness skin transplantation due to the existence of granulation wounds. After medium thick skin transplantation, the healing barrier of donor site will be caused, resulting in the generation of new surface. Thick blade skin transplantation can solve the problem of the low survival rate. However, due to the lack of dermis after skin grafting, the friction resistance and pressure resistance of the surface are poor, which is easy to cause secondary rupture. In this study, acellular allogeneic dermal matrix and autologous skin combined with skin grafting for wound repair can overcome the above problems in DF patients [20]. MRI has great advantages in distinguishing various types of soft tissue infection and distinguishing between tissue and bone marrow. It can detect abnormal bone marrow signals early and accurately identify the range of soft tissue infection. Therefore, MRI can be used as an important means for routine diagnostic examination and posttreatment efficacy evaluation of DF to help optimize and improve the quality of life of patients with DF [24].

A total of 78 DF patients were selected as research subjects and divided into the experimental group (composite skin graft) and control group (autologous skin graft). MRI scanning was performed before and after treatment to compare the changes of MRI signal sequence intensity and other image data characteristics of patients, as well as the changes of experimental observation indicators such as healing time, recurrence rate, and scar score. This study aimed to analyze the application value of MRI image data features based on the deep learning algorithm in evaluating the treatment of DF with compound skin graft. The results showed that there were no substantial differences in age, gender, course of disease, body mass index, HbAlC, and Wagner grading between the two groups (*P* > 0.05), which increased the comparability of MRI image data in the evaluation of treatment efficacy between the two groups after treatment. The comparison analysis of the scanning sequence signal intensity of patients obtained by MRI scan before and after treatment showed that the T1WI signal intensity of the experimental group was considerably increased after treatment, while the signal intensity of fat-suppressed T2WI and fat-suppressed T1WI enhanced sequence was considerably decreased (*P* < 0.05). This indicated that there were differences in the intensity of MRI scan sequence T1WI, fat-suppressed T2WI, and fat-suppressed T1WI enhancement sequence before and after treatment, which were closely related to the treatment effect. Compared with the control group, there was no statistical difference in the wound healing time and complete healing rate of the experimental group (*P* < 0.05), while the recurrence rate, healing time of the donor skin area, and scar score were considerably decreased (*P* < 0.05). This was consistent with the research results of Campitiello et al. [25]. After acellular treatment, the composite skin was fused with the body, resulting in the formation of epidermis and basement membrane, complete dermis structure, and less infiltration of inflammatory cells, which did not affect normal wound healing. Lantis et al. [26] also pointed out that due to DF end blood supply obstacles and factors of local high sugar, the recurrence rate was high, and the integrity of the skin was restored after transplantation of the composite skin, promoting capillary and normal expression of growth factors and cytokines and improving local microvascular environment, so the recurrence rate was also decreased. Through calculation of accuracy, specificity, and sensitivity, it was found that MRI imaging information had high accuracy, specificity, and sensitivity in evaluating the therapeutic effect of DF patients, which were 85.2%, 89.75%, and 86.47%, respectively. The specificity and sensitivity of the therapeutic effect of DF were evaluated according to MRI imaging information, and ROC curve was plotted. AUC was determined to be 0.838 according to ROC, indicating that the characteristics of MRI image data can provide a reference for the evaluation of the therapeutic effect after compound skin transplantation for DF. Some studies evaluated the correlation between diagnosis and treatment performance of DF image MRI and laboratory examination. It was found that MRI could be used to monitor and evaluate the curative effect of treating DF. As a noninvasive monitoring method, it is simple to operate and very sensitive and accurate to the pathological changes of DF patients, which is consistent with the results of this study [27]. In short, MRI image data features based on the deep learning algorithm can provide auxiliary information for the efficacy evaluation of compound skin transplantation for DF, which has a great application value.

## 5. Conclusion

In this study, DF patients in the experimental group and the control group were treated with compound skin graft and autologous skin graft, respectively. MRI was used to compare the signal sequence intensity, clinical healing time, recurrence rate, scar score, and other indicators of the two groups. The results showed that T1WI, fat-inhibited T2WI, and enhanced sequence signal intensity of MRI scan were correlated with the therapeutic effect. The accuracy, specificity, and sensitivity of MRI image data characteristics to evaluate the therapeutic effect of diabetic foot were high, which could provide a reference for the evaluation of the therapeutic effect of DF after compound skin transplantation. The deficiency of the study is that the sample size is small, which is relatively single, and does not have randomness and wide applicability. In the future study, multisite, multitype, and large sample size analysis and research will be considered. In conclusion, this work provides some reference for the treatment of diabetic foot transplantation.

## Figures and Tables

**Figure 1:** MRI scanning parameters. (a) The repetition time of each scan sequence. (b) The echo time of each scan sequence. (c) The length of echo chain of each scan sequence.

**Figure 2:** SSD detection flowchart.

**Figure 3:** MRI images of different DF patients.

**Figure 4:** SSD target detection.

**Figure 5:** Comparison of basic data between the two groups. (a) The comparison results of gender ratio, HbAlC, body mass index, and disease course between the two groups. (b) The comparison results of average age and proportion of patients in Wagner classification between the two groups.

**Figure 6:** Changes in MRI sequence signal intensity before and after treatment. ^*∗*^Substantial difference, *P* < 0.05.

**Figure 7:** Comparison of wound healing time and donor site healing time between the two groups after treatment. ^*∗*^Substantial difference, *P* < 0.05.

**Figure 8:** Comparison of complete healing rate, recurrence rate, and scar score between the two groups after treatment. ^*∗*^Substantial difference, *P* < 0.05.

**Figure 9:** ROC curve results of MRI image data characteristics.

## Data Availability

The data used to support the findings of this study are available from the corresponding author upon request.
